# Regulation of Human Innate Lymphoid Cells in the Context of Mucosal Inflammation

**DOI:** 10.3389/fimmu.2020.01062

**Published:** 2020-06-23

**Authors:** Anja Schulz-Kuhnt, Stefan Wirtz, Markus F. Neurath, Imke Atreya

**Affiliations:** Department of Medicine 1, University Hospital of Erlangen, Erlangen, Germany

**Keywords:** innate lymphoid cells, mucosal inflammation, human immune system, cytokine, ILC plasticity, tissue migration

## Abstract

Since their identification as a unique cell population, innate lymphoid cells (ILCs) have revolutionized our understanding of immune responses, leaving their impact on multiple inflammatory and fibrotic pathologies without doubt. Thus, a tightly controlled regulation of local ILC numbers and their activity is of crucial importance. Even though this has been extensively studied in murine ILCs in the last few years, our knowledge of human ILCs is still lagging behind. Our review article will therefore summarize recent insights into the function of human ILCs and will particularly focus on their regulation under inflammatory conditions. The quality and intensity of ILC involvement into local immune responses at mucosal sites of the human body can potentially be modulated via three different axes: (1) activation of tissue-resident mature ILCs, (2) plasticity and local transdifferentiation of specific ILC subsets, and (3) tissue migration and accumulation of peripheral ILCs. Despite a still ongoing scientific effort in this field, already existing data on the fate of human ILCs under different pathologic conditions clearly indicate that all three of these mechanisms are of relevance for the clinical course of chronic inflammatory and autoimmune diseases and might likewise provide new target structures for future therapeutic strategies.

## Introduction

Having been overlooked for ages, helper innate lymphoid cells (ILCs) have been increasingly recognized as key immunological players since their discovery as a distinct cell population in 2010 (1–3). Since then, as a result of an immense amount of scientific effort, a prominent role has been assigned to ILCs as initiators and amplifiers of protective but also detrimental immune responses in various tissues, making them interesting potential therapeutic targets (4, 5).

Phenotypically, ILCs are classified as lymphoid cells that lack the expression of lineage markers defining any known lymphoid or myeloid cell population (6). Functionally, ILCs share core effector features with T cells, even though they are characterized by a lack of rearranged antigen-specific receptor expression. This enables full activation of ILCs independent from the antigen-presentation and -recognition machinery and thereby the induction of rapid immune responses (7). After their stepwise development from a common lymphoid progenitor cell [reviewed elsewhere (8–10)], mature ILCs can be categorized into three main subgroups by analogy to T cells, based on their dependency on transcription factors and the secretion of effector cytokines: type-1, type-2, and type-3 ILCs (ILC1s, ILC2s, and ILC3s, respectively) (11). ILC1s can be further subdivided into cytotoxic NK cells and helper ILC1s (12). Whereas, classic NK cells are well-known to mediate a potent cytolytic effector function and have been extensively studied and reviewed already (13, 14), this review will focus on helper ILCs in particular. While helper ILC1s critically depend on the transcription factor T-bet and are able to amplify immune responses against intracellular pathogens via an extensive release of IFN-γ and TNF-α (15, 16), ILC2 function is regulated by GATA-3 and RORα as key transcription factors, and the effector cytokines IL-5, IL-13, IL-9, and IL-4 relevantly impact the resolution of helminth infections (6, 17, 18). Finally, analogous to type-17 T helper (Th17) cells, RORγt represents the master transcription factor of ILC3s, including lymphoid tissue inducer (LTi) cells as well as non-LTi ILC3 subsets. While LTi cells play a particular role in lymphoid organogenesis, ILC3s in general are characterized by the secretion of IL-17A, IL-22, and GM-CSF and are thereby involved in the immunological control of extracellular microbes (19–21). In addition to these three classical subgroups, in analogy to regulatory T cells (Tregs), regulatory ILCs (ILCregs) were recently identified in the intestine that suppressed ILC1s and ILC3s in an IL-10-dependent manner, while TGF-β served as autocrine growth factor (22).

Helper ILCs are primarily located in close proximity to mucosal barriers, like the pulmonary (23) and intestinal epithelium (19), which are highly prone to environmentally driven tissue damage and pathogen entry. There, ILCs are involved in the first line of immune response via the instant release of extraordinary amounts of effector cytokines that orchestrate further immune reactions (24, 25). However, tight control of local ILC numbers and their activation status is crucial to guarantee barrier integrity and tissue homeostasis without the induction of overwhelming and chronic immune responses.

Based on their overall low frequency and redundant functions with T helper (Th) cells as well as the finding that ILC deficiencies appeared to be asymptomatic in humans with competent adaptive immune cells, ILCs were suggested to be expandable under natural conditions. This assumption, however, was only based on a small cohort living under modern hygiene and medical standards (26) and does not seem to hold true under pathological conditions. In severe liver fibrosis, for example, local ILC2 frequencies were exclusively increased while the proportion of Th2 cells was unaltered (27), indicating a particular role for ILCs during fibrotic tissue remodeling. In line with this, a cell-specific regulation and thus activation profile of ILCs and Th cells has been described. ILC2s, for instance, rely on DR3 and IL-9R signaling for activity and survival, which was not the case in Th cells (28, 29). On a functional level, it was particularly the CD3^−^ lamina propria mononuclear cell (LPMC) fraction that showed significantly increased IL-22 production in inflammatory bowel disease (IBD) patients compared to controls but not Th cells (30), assigning ILCs a distinct and important effector role in disease. Moreover, the rapid availability of effector cytokines and the finding that ILC2s are more potent in the production of IL-5 and IL-13 than are CD4^+^ T cells in blood and sputum of patients suffering from severe asthma (31) distinguishes ILCs from Th cells, making them a functionally unique cell population. Importantly, ILC activity has been shown to be crucial for efficient T cell responses under various conditions (32–34), demonstrating their far-reaching influence on efficient immunity.

And while ILCs have been shown to be involved in many different immunological phenomena, including host protection, wound healing, anti-tumor immune responses, autoimmunity, graft-vs.-host reaction, chronic inflammation, and fibrosis in numerous murine studies (35–41), the transfer of these findings into the human system and a related functional characterization of ILCs in the context of human disease still remains incomplete. Even though murine and human ILCs share basic characteristics, human ILCs have been shown to markedly differ in several key aspects from their murine counterparts (8, 42, 43), making translational research on human ILCs inevitable. The first important hints of the existence of species-specific ILC biology arose from studies that described variances in the ILC surface marker profile between mice and men. Regarding ILC1s, a distinct subset restricted to an intraepithelial localization and producing IFN-γ in response to IL-12 and IL-15 was described that differs in its αE integrin and NKp44 expression between mice and humans (44, 45). Similarly, two distinct functional subtypes of ILC2s, namely inflammatory and natural ILC2s, could be identified in both species but differed in their surface maker profiles. While, in mice, these subtypes were distinguished by ST2 and KLRG1 expression (46), functionally similar subtypes in humans were rather discriminated by their c-Kit expression (47). In the group of ILC3s, two subtypes secreting mainly IL-22 or IL-17 have been described in varying proportions and with altered marker expression in the two species (45, 48). These phenotypical and numerical differences strongly imply that the localization and activation of murine and human ILCs might also be partly regulated by separate molecular mechanisms. And indeed, on a functional level, there is an ongoing and controversial discussion as to whether ILCs of the two species follow the same mechanistic concept of tissue distribution and maturation in adulthood. While parabiosis experiments in mice strongly suggested that ILCs have a tissue-resident, long-lived nature and mostly excluded their recirculation and organ redistribution upon acute inflammation (49, 50), a very recent study postulated a concept of circulating uni- and pluripotent human ILC precursors that are able to migrate into tissue and undergo final differentiation in response to local environmental signals (51). This permanent presence of ILC precursors in the peripheral blood together with the idea of tissue ILC differentiation (51) is in accordance with the well-described phenomenon of a significant organ accumulation of defined ILC subsets in the context of inflammatory tissue injury. Indeed, patients suffering from IBD show distinct numerical alterations in the ILC composition in the intestinal mucosa that depend on disease duration (15, 52, 53). Moreover, atopic dermatitis, hepatic fibrosis, and chronic rhinosinusitis are associated with an accumulation of ILC2s in skin, liver, and sinonasal tissue, respectively (23, 27, 54). This association strengthens the clinical urgency of directly analyzing human ILCs, especially since most murine studies are biased by the use of specific-pathogen-free or immunodeficient mice without a functional adaptive immune system that do not sufficiently represent the human situation and might therefore not allow results to be directly translated into the human system (6).

The following review article will therefore summarize recent insights into the function of human helper ILCs and will focus on their regulation at mucosal sites under inflammatory conditions in particular. The quality and intensity of ILC-driven local immune responses at mucosal tissues can be modulated via the activation status as well as a numerical regulation of local ILCs (Figure 1). This potentially involves three different axes: (1) activation or inhibition of tissue-resident ILCs, (2) numerical regulation of mature local ILCs via cell death, proliferation, or differentiation from local precursors or other ILC subsets, and (3) tissue-specific migration and regional accumulation of peripheral ILCs (12, 15, 35, 51, 55). Despite ongoing scientific efforts in this field, already existing data on the fate of human ILCs under various pathological conditions clearly indicate that all three mechanisms relevantly impact the clinical course of chronic inflammatory and autoimmune diseases and might therefore provide new target structures for future therapeutic strategies.

**Figure 1:** Mechanisms regulating local ILC activity. To adapt ILC functions at mucosal barriers to the respective environmental need, local ILC numbers and their activity can be regulated by soluble mediators or direct cell-cell interactions (green background). To date, cytokines and lipid mediators represent the most commonly described soluble regulators of human ILCs and can be released, for instance, by stress-sensing epithelial cells or other immune cells like mast cells. Furthermore, neurotransmitters and neuropeptides have also been suggested to directly interact with ILCs. In addition, cell-cell contact-dependent regulation of ILCs is based on their interaction with endothelial, stromal, and other immune cells. Upon sensing these signals, ILC activity (orange background) and their local number (yellow background) can be controlled. Tissue ILC counts can be modulated directly by cell death and proliferation or the differentiation of local ILC precursors into mature cells. Moreover, ILCs are plastic cells, enabling the transdifferentiation of one subset into another. Altered local ILC numbers can additionally result from the migration of ILCs either within an organ or from/to a distal site. Representatively, regulators modulating ILC activities on various levels are shown. *In vivo*, multiple mechanisms controlling local ILC activity are likely to act synergistically, enabling the activation or suppression of ILC activities in a highly controlled fashion. However, dysbalanced and overwhelming ILC responses are often unable to successfully fight pathogens or can even trigger inflammatory diseases.

## Regulation of Human ILCs

### Helper ILCs as Guardians at Mucosal Barriers

Forming large surfaces with the body's outer environment, mucosal tissues, including the respiratory, gastrointestinal (GI), and urogenital tract, have to guarantee stable protection against invading pathogens and various harmful substances. Therefore, the maintenance of epithelial integrity as a physical barrier and the capacity to initiate immediate but controlled mucosal immune responses are essential. Based on their instant, antigen-independent ability to secrete effector cytokines, ILCs represent ideal guardians in mucosal tissues. In line with this, ILCs have been shown to preferentially accumulate in organs with mucosal barriers in close proximity to the epithelium (56, 57).

From the esophagus to the colon, all helper ILC subsets have been described in the human GI tract, with the highest frequencies of total helper ILCs residing in the intestine (58). While ILC1s appeared to be enriched in the human gingivae (59) and esophagus (58), NKp44/NCR^+^ ILC3s represent the most abundant subtype in the gut (53, 55, 58), suggesting an important function for ILC3s in intestinal homeostasis. In contrast, only low frequencies of ILC2s have been detected in both the upper and lower GI tract (53, 55, 58, 60). Under chronic inflammatory conditions, the local ILC composition is drastically altered in inflamed areas (53), as shown by the distribution of intestinal ILCs in IBD patients (15, 30, 52, 53). Indeed, altered numbers of colonic NKp44^+^ ILC3s have been described already in early in IBD (15), and IL-22 production by ileal ILCs was shown to be increased in patients with mild or moderate CD (30). In accordance with the common concept that the immunopathogenesis of CD and UC is dominated by type-1 and type-2 immunity, respectively (61), CD patients were also characterized by increased ILC1 frequencies (15, 53) as well as IL-17-secreting ILCs (52), whereas UC patients displayed increased proportions of ILC2s during the course of disease (53). Interestingly, ILCregs were described in the murine and human gut as well, likely serving as a control mechanism to suppress exaggerated immune responses (22). Overall, these disease-dependent alterations of ILC frequencies in the human intestine suggest defined functions of ILC subgroups under specific inflammatory conditions and at different anatomical sites, implicating a milieu-dependent fine-tuning of each subset.

In the respiratory tract, research has focused on the ILC2 subset in particular, given the pivotal role of type-2 mediated immunity in allergic airway diseases (62). Nevertheless, all three helper ILC subsets have been described in lung tissue, with ILC2s and ILC3s being most abundant (55, 60, 63). During adulthood, several disorders associated with acute and chronic inflammation of the lung are characterized by altered ILC frequencies. For instance, asthmatic patients showed increased ILC2 frequencies and effector cytokines in peripheral blood, sputum, and bronchoalveolar lavage (BAL), which turned out to correlate with the severity of clinical symptoms (31, 64–68). Next to this allergic context, lung inflammation resulting from infection with *Mycobacterium tuberculosis* was characterized by reduced blood pools of albeit activated ILC1s, ILC2s, and ILC3s and a corresponding accumulation of these cells in the infected lung tissue (69). The observations that ILC2s were enriched in the BAL of patients with idiopathic pulmonary fibrosis (37) and that the destructed lung tissue of patients with chronic obstructive pulmonary disease (COPD) showed elevated local ILC1 and NKp44^−^ ILC3 frequencies at the expense of ILC2s (55) point to a potential reciprocal interference between pulmonary ILCs and fibrotic tissue remodeling. Furthermore, ILC2s are present in nasal tissue, where they also showed increased proportions upon upper airway inflammation, such as for example, in patients suffering from allergic rhinitis (70, 71) and chronic rhinosinusitis with nasal polyps (55, 60, 72). Contrarily, nasal polyps in the context of cystic fibrosis were dominated by enhanced percentages of NKp44^−^ ILC3s (72). These findings indicate that various helper ILC subsets play a key role in inherited as well as allergen-, bacterial-, and environmental-driven inflammatory lung disorders. Nevertheless, inconsistent study designs and patient and control cohorts, as well as variable marker combinations defining ILC subsets, led to partly controversial results (64, 70, 71) and impede larger meta-analyses. Based on the current pandemic situation induced by the new coronavirus, SARS-CoV-2, the question of an ILC involvement in the resulting lung disease, COVID-19, is being raised. Indeed, there are good grounds for speculating about a relevant disease-modulating capacity of mucosal ILCs in this viral infection: ILCs are present in the lung tissue even under steady-state conditions (55, 60, 63) and are located in direct proximity to the respiratory epithelium (57) and thus to ACE2-expressing pneumocytes, which have been described as the predominant entry and replication site of SARS-CoV-2 (73). Accordingly, diffuse alveolar damage, as detected histologically in lung biopsies of COVID-19 patients (74), represents a well-described trigger of local ILC activation, classically resulting in the initiation and regulation of far-reaching immune responses (75). Besides epithelial cell-derived alarmins, the activation status of ILCs could also be influenced by immune cell-secreted cytokines upregulated in the course of severe COVID-19 (76, 77), such as IL-6 (stimulatory effect on human ILC3s) or IL-10 (inhibitory effect on ILC2s) (see also Table 1). Thus, on a functional level, a relevant contribution of activated pulmonary ILCs to the anti-viral immune response and to the consolidation of epithelial damage can be expected and might mainly be relayed via an excessive release of ILC-derived cytokines. And indeed, altered NK cell frequencies in COVID-19 patients (109) have been the first proof that infection with SARS-CoV-2 does modulate the ILC compartment. Especially in severe COVID-19 cases, NK cell percentages turned out to be downregulated in line with the overall observed lymphocytopenia (109, 110). However, upon recovery, restoration of NK cell frequencies has been described (109, 110), implicating a relevant function for NK cells in the resolution of this viral infection. In general, NK cells, together with helper ILC1s, are considered to be important effector cells, fighting various viral diseases and representing an early source of IFN-γ and TNF-α (111, 112), with the latter being highly upregulated in the plasma of COVID-19 patients (113). Moreover, data acquired in the murine system indicated that pulmonary ILC2s promoted IgM production in B cells and thus supported early humoral immunity directed against respiratory antigens (114). As a morphological indicator of an ongoing consolidation of epithelial injury, lung tissue of COVID-19 patients could be characterized by an accumulation of fibrin in the alveolar wall and airspaces (74). Of note, pulmonary ILC2s and the ILC2-released cytokine IL-13 have been described as potent mediators of collagen deposition, at least in murine models of lung fibrosis (37). In addition, based on analyses in a mouse model of influenza virus infection, ILC2-derived AREG was postulated to protect and restore the airway epithelium upon viral damage (115). Besides the potential involvement of ILCs in the anti-viral immune response directed against SARS-CoV-2, it should also be taken into account that, at least compared to other immune cell fractions, murine ILCs, and especially ST2-negative ILC2s derived from the small intestine, appeared to show a relatively high expression of the SARS-CoV-2 entry receptor ACE2 at the RNA level (116). It will thus be interesting to clarify in future studies whether ILCs might represent a cellular target for SARS-CoV-2 infection and potentially even virus replication. Since an enormous amount of scientific effort is being exerted worldwide to further decipher the pathology of COVID-19, we can expect to achieve improved and more concrete insights into the functional role and potential therapeutic targeting of local ILC pools during the clinical manifestation and/or exacerbation of this threatening and fast-spreading disease very soon.

**Table 1:** Local regulators of ILC activity.

**ILC subgroup**	**Regulator**	**Class**	**Regulation**	**ILC origin**	**Pathophysiological context**	**References**
ILC1	IL-12	Cytokine	+	Tonsils, peripheral blood	Immunity to mycobacteria, CD	(15, 44, 55, 78)
ILC1	IL-15	Cytokine	+	Tonsils	CD	(44)
ILC1	IL-18	Cytokine	+	Intestine	Commensal and pathogenic gut microbiota	(79)
ILC1	IL-1β	Cytokine	+	Intestine	Commensal and pathogenic gut microbiota	(79)
ILC1	TGF-β	Cytokine	–	Peripheral blood	IBD	(80)
ILC2	IL-33	Cytokine	+	Peripheral blood; nasal polyps, fetal gut, tonsils	IBD, asthma	(18, 55, 60, 68, 81)
ILC2	IL-25	Cytokine	+	Peripheral blood; nasal polyps, fetal gut, tonsils	IBD, asthma	(18, 60, 68, 81)
ILC2	TSLP	Cytokine	+	Peripheral blood; nasal polyps, fetal gut, tonsils	Chronic rhinosinusitis with nasal polyps, IBD, asthma	(18, 55, 60, 81)
ILC2	IL-1α/β	Cytokine	+	Peripheral blood, tonsils	IBD, COPD	(55, 60, 82)
ILC2	IL-18	Cytokine	+	Peripheral blood	Inflammatory cutaneous diseases	(12)
ILC2	TL1A	Cytokine	+	Peripheral blood	Helminth infection, type-2 lung inflammation	(28)
ILC2	IL-4	Cytokine	+	Peripheral blood	Chronic rhinosinusitis with nasal polyps	(55)
ILC2	IL-10	Cytokine	–	Peripheral blood, nasal polyps	Grass polen immunotherapy	(80, 83)
ILC2	TGF-β	Cytokine	–	Peripheral blood, nasal polyps	Grass polen immunotherapy	(83)
ILC2	IFN-α	Cytokine	–	Peripheral blood	Suppression of airway inflammation	(84)
ILC2	IFN-β	Cytokine	–	Cord blood	Asthma	(85)
ILC2	CCL1	Cytokine	+	Peripheral blood	Anti-helminth and - parasitic immunity	(86)
ILC2	PGD_2_	Lipid mediator	+	Skin, peripheral blood	Allergy	(87, 88)
ILC2	LTE_4_	Lipid mediator	+	Peripheral blood	Atopic dermatitis	(89)
ILC2	PGI_2_	Lipid mediator	–	Peripheral blood	Allergen-induced lung inflammation	(90)
ILC2	PGE_2_	Lipid mediator	–	Peripheral blood, tonsils	Allergic lung inflammation	(91)
ILC2	Lipoxin A4	Lipid mediator	–	Peripheral blood	Asthma	(88)
ILC2	Retinoic acid	Vitamin	+	Peripheral blood	Allergic inflammation	(92)
ILC2	1,25D	Vitamin	–	Peripheral blood	Allergic inflammation	(92)
ILC2	ICAM-1–LFA-1	ILC2–immune cell interaction	+	Peripheral blood	IL-33-induced lung inflammation	(93)
ILC2	GITR–GITR-L	ILC2—immune cell interaction	+	Peripheral blood	Allergic lung inflammation	(94)
ILC2	RANK-RANK-L	ILC2–immune cell interaction	+	Peripheral blood, nasal polyps	Chronic rhinosinusitis with nasal polyps	(95)
ILC2	ICOS–ICOS-L	ILC2 –ILC2	+	Peripheral blood	IL-33-induced airway hyperreactivity	(96)
ILC2	ICOS–ICOS-L	ILC2 –iTreg	–	Peripheral blood	Resolution of airway inflammation	(97)
ILC2	MHCII–TCR	ILC2–Th cell	+	Peripheral blood	Helminth infection	(34)
ILC2	NKp30—B7-H3	ILC2–keratinocytes	+	Peripheral blood	Atopic dermatitis	(98)
ILC2	KLRG1–E cadherin	ILC2–endothelial cell	–	Skin	Atopic dermatitis	(54)
ILC2	PD-1	Checkpoint inhibitor	–	Peripheral blood	Helminth infection	(99)
ILC3	IL-23	Cytokine	+	Intestine	IBD	(30, 52)
ILC3	IL-1β	Cytokine	+	Intestine	IBD	(30)
ILC3	IL-18	Cytokine	+	Tonsils	Maintenance of tissue integrity	(100)
ILC3	IL-15	Cytokine	+	Tonsils	Maintenance of tissue integrity	(100)
ILC3	IL-6	Cytokine	+	Colon	IBD	(101)
ILC3	TL1A	Cytokine	+	Intestine, tonsils, hematopoietic stem cell-derived	IBD	(30, 102)
ILC3	IFN-α	Cytokine	–	Tonsils	N/A	(100)
ILC3	IFN-γ	Cytokine	–	Tonsils	N/A	(100)
ILC3	TLR2 ligand	Bacterial metabolite	+	Tonsils	N/A	(103)
ILC3	AHR receptor	Bacterial metabolite	+	Tonsils, intestine	*C. rodentium* infection	(104, 105)
ILC3	Bacillus anthracis toxin	Bacterial metabolite	–	Tonsils	Anthrax	(106)
ILC3	Acetylcholin	Neurotransmitter	+	Peripheral blood	Resolution of *E. coli* infection	(107)
ILC3	1,25D	Vitamin	+/–	Tonsils, intestine	IBD	(108)

*CD, Crohn's disease; IBD, Inflammatory bowel disease; COPD, Chronic obstructive pulmonary disease*.

Although ILCs have been extensively studied in the lung and gut over the last decade, little is known about their role at the mucosal surface of the urogenital tract. So far, helper ILCs have been analyzed in the uterus and decidua only during pregnancy, and here they were suggested to be important effectors initiating tissue remodeling during implantation (48). In particular, ILC3s and ILC1s were described to be involved in the maintenance of early pregnancy (117, 118). Increased frequencies of ILC3s and ILC2s, however, were associated with overwhelming inflammation in preterm labor (119). In order to further validate the functional relevance of ILCs in this context, it will be of crucial importance to gain more detailed insights into the potential underlying ILC-driven effector mechanisms and molecular mediators.

Collectively, extensive work on the role of helper ILCs at mucosal barrier sites in humans has revealed clear associations of defined ILC subsets with various inflammatory and fibrotic diseases. However, some important questions remain not fully answered: are altered ILC frequencies are a cause or consequence of the associated tissue pathology and which molecular mechanisms underlie their numerical and functional regulation?

### Local Modulators of ILC Activity

#### Local Regulation of Human Helper ILC1s

On the one hand, helper ILC1s have been suggested to be important effector cells that fight intracellular pathogens and bacteria in order to maintain tissue homeostasis. On the other hand, altered ILC1 frequencies in CD (15, 53) and COPD patients (55) indicate the involvement of this ILC subtype in chronic inflammation. Careful regulation of ILC1 activity is thus strictly required to allow the secretion of protective effector cytokines but, at the same time, prevent sustained and overwhelming immune activation resulting in pathologic tissue remodeling and chronic injury.

Cytokines represent one of the main regulatory stimuli of innate immune responses (120). In the case of human ILC1s, the pro-inflammatory cytokine IL-12, which has already been well-known for its ability to promote type-1 immune responses (121), turned out to be also of immense importance for the activation of ILC1s and subsequent IFN-γ release (15, 78) as shown in primary human ILC1s purified from tonsils and peripheral blood (15, 78). In accordance with this, ILC1s expressed higher mRNA levels of the IL-12 receptor subunit B2 (IL12-RB2) than ILC2s and ILC3s (15, 55). Especially in combination with IL-2 and/or IL-18, IL-12 was identified as a potent inducer of IFN-γ production in *in vitro* cultured human ILC1s (15, 55). This IL-12 responsiveness was also true for the unique subset of intraepithelial human NKp44^+^CD103^+^ ILC1s, which have been suggested to mirror key cytotoxic features of tissue-resident CD8^+^ memory (Trm) cells (44, 122). While IL-18 failed to synergize with IL-12 in the induction of NKp44^+^CD103^+^ ILC1-derived IFN-γ production, IL-15 alone and in combination with IL-12 served as an effective stimulus (44). As the main cellular source of IL-12, antigen-presenting cells (APCs) release high amounts of this type-1 cytokine after exposure to bacteria (123). This is of particular relevance in the context of IBD, where intestinal barrier defects lead to increased mucosal infiltration of luminal bacteria (124). In response to the enhanced release of IL-12p70, IL-18, and IL-1β by local myeloid dendritic cells (DCs), intestinal ILC1s are able to secrete increased levels of the pro-inflammatory cytokines IFN-γ and TNF-α and thus relevantly support the mucosal immune response against bacterial intruders. This was true for gram-negative commensals and pathogens, e.g., *Acinetobacter junii* and *Salmonella typhimurium*, as shown in *in vitro* co-cultures of human ILC1s and lamina propria mononuclear cells (LPMCs) (79). Without proper regulation of this response, chronic inflammation can be established. In CD patients, for example, LPMCs showed hyperresponsiveness toward bacterial components, resulting in enhanced IL-12 levels (125, 126), which was associated with increased accumulation of IFN-γ-expressing ILC1s in the inflamed mucosa (15, 53). Besides monocytes and DCs, co-culture experiments demonstrated that epithelial cells were also able to translate luminal danger signals, such as TLR2, into a stimulatory trigger for human intraepithelial NKp44^+^CD103^+^ ILC1s to produce IFN-γ. Thus, efficient pathogen-mediated activation of intraepithelial ILC1s might even occur in the absence of epithelial barrier destruction (44). To control this, TGF-β was identified as a negative regulator of ILC1-mediated IFN-γ, but not TNF-α secretion (80), a mechanism dysregulated in IBD patients (127).

In addition to the here-described stimuli (summarized in Table 1), human blood or tissue ILC1s have been shown to express further surface receptors, such as IL-4R, IL-9R, and ICOS (55), that potentially transmit regulatory signals. This, however, still has to be validated functionally for human ILC1s, and further research will thus be necessary to fully decipher the mechanisms regulating ILC1 activity in humans.

#### Local Regulation of Human Helper ILC2s

ILC2s and their role in physiological and pathological processes have been extensively studied (128–131). Based on analyses in the murine system, local ILC2s represent an unusually long-lived cell type (132), which therefore requires tightly controlled effector functions. A complex network regulating the activity of tissue-resident ILC2s has been identified (summarized in Table 1). This includes soluble mediators, such as cytokines and lipid mediators, as well as direct cell-cell interactions.

##### Soluble modulators of human ILC2s

Among numerous cytokines, the alarmins IL-25, IL-33, and thymic stromal lymphopoietin (TLSP) constitute the central activation unit of ILC2s (18, 55, 60, 68, 81). It is noteworthy that cytokine-mediated ILC2 activation was accompanied by elevated receptor expression of ST2, IL17BR, and TSLPR on the cell surface, enabling alarmins to further potentiate their stimulatory effects (81). Successful *in vitro* stimulation of human ILC2s was reflected in characteristic morphological alterations, an activated phenotype (68), and increased survival and proliferation of stimulated ILC2s (81). Probably most relevant, stimulated ILC2s showed enhanced effector functions in the form of the secretion of large amounts of type-2 effector cytokines, including, primarily, IL-13 and IL-5, but also IL-4 and GM-CSF (18, 55, 60, 68, 81). In multiple *in vitro* stimulation experiments with primary human ILC2s and stable ILC2 cell lines, combinations of multiple cytokines turned out to induce ILC2 activation most potently. Interestingly, TSLP alone or in combination with IL-25 and IL-33 harbored the highest pro-survival capacity (81), whereas IL-33 appeared to be an important co-factor for the induction of ILC2 proliferation in different cytokine combinations (81). Regarding the effector functions, several studies reported that IL-25, IL-33, and TSLP alone had no or only suboptimal effects on the secretion of selected effector cytokines (18, 60, 82, 92) but displayed synergistic effects with IL-2 (18, 81) or in combination with each other (54, 68, 81). IL-2 is well-known for its pro-survival effects on lymphoid cells; however, it represents a sufficient ILC2 stimulus only in the presence of synergistic co-factors (18, 55, 68, 81, 82). Several studies indicated that the combined effects of IL-25, IL-33, TSLP, and IL-2 represented the most potent stimuli for ILC2 activation (18, 60, 68, 81) and might also resemble the *in vivo* situation very closely. In line with the role of ILC2s as early mediators of mucosal defense, epithelial cells responding to stress signals represent very prominent local sources of the alarmins IL-25, IL-33, and TSLP (133). For example, in patients suffering from chronic rhinosinusitis, nasal polyp epithelial cells expressed TSLP, which directly activated local ILC2s (18). Besides the epithelium, relevant expression of alarmins could also be detected in endothelial cells, Th2 cells, mast cells, fibroblasts, and macrophages (134–139). So far, most human studies have been conducted with peripheral blood ILC2s. However, tissue-resident ILC2s derived from nasal polyps (18), fetal gut (60), and tonsils (82) showed a similar activation behavior. Further evidence comes from murine experiments showing the ability of IL-33 and IL-25 to boost ILC2 responses *in vivo* (131).

While most of the common ILC2 activators, like IL-33, IL-25, and TSLP, belong to the group of epithelial-derived alarmins and are released upon various stress conditions, IL-1β represents an inflammasome-dependent pro-inflammatory cytokine well-known to trigger fever and the mobilization of neutrophils (140, 141). Although an ILC-activating effect of IL-1β has first been described for the ILC3 compartment (142), marked expression of the IL-1β receptor and respective IL-1β responsiveness were also observed in human ILC2s (55, 60). At least in experiments performed *ex vivo*, IL-1β and IL-1α together with IL-2 served as potent stimuli for human blood ILC2 proliferation and the production of IL-5 and IL-13 (55, 81, 82). In addition, IL-1β was shown to increase the expression of ST2L, IL-17RB, and, to a lesser extent, TSLPR on human ILC2s (82), which was suggested to be a priming signal enhancing the effect of epithelial cell-derived alarmins and explaining their additive effect (82). However, as further discussed later in this article (see paragraph on ILC Plasticity and Tissue Differentiation), other studies indicated that IL-1β might support ILC2-to-ILC1 plasticity (82). Within tissues, activated IL-1β is mainly released by macrophages, DCs, and neutrophils, classically after exposure to Toll-like receptor ligands or DAMP (141), and increased levels of this cytokine could be observed in the lungs of COPD patients, in the inflamed intestinal mucosa of IBD patients and in lesions of autoimmune and inflammatory skin diseases (143–145).

*In vitro* stimulation with the pro-inflammatory cytokine IL-18 could additionally induce cytokine secretion in human blood ILC2s via the IL-18R (146). Interestingly, in mice, a skin ILC2 subset was identified to preferentially respond to IL-18. These data clearly pointed to the existence of tissue-specific ILC subsets with unique receptor profiles and thus distinct abilities to respond to environmental stimuli (147). In line with this, IL-18 is thought to be involved in various inflammatory cutaneous diseases, including atopic dermatitis (148), suggesting a potential role for active ILC2s in these diseases as well.

The TNF superfamily member TL1A has been suggested as another potent activator of human ILC2s that express high levels of its receptor DR3 (death receptor 3; TNFRSF25) (28). Primarily secreted by alarmed epithelial, endothelial, and myeloid cells, TL1A induced effector cytokine secretion by human ILC2s and acted additively to IL-25 or IL-33 *in vitro*. Murine *in vivo* experiments further revealed the functional importance of this TL1A-driven ILC2 activation in regulating helminth infections and driving type-2 lung inflammation (28).

In combination with external stimulation, IL-4 (55) and IL-9 (29, 149) have been suggested to further boost proliferation and cytokine secretion of activated ILC2s in an autocrine fashion. In the case of IL-4, this autocrine loop could be functionally proven in *ex vivo* stimulated human blood ILC2s (55). Regarding IL-9, the direct functional proof is still restricted to murine data showing the importance of IL-9-driven ILC2 stimulation for the maintenance of lung homeostasis (29, 150) as well as for the resolution of arthritis (149). In accordance with the latter, association data from patients with rheumatoid arthritis showed an inverse correlation between blood ILC2 counts and disease activity (149). Moreover, the chemokine CCL1 could recently be identified as another autocrine activator of ILC2 function in mice and men, mediating its effects via CCR8 signaling (86).

In order to dampen overwhelming ILC2 activity, negative regulators are inevitable to guarantee controlled immune responses. However, our understanding of those immunological mechanisms limiting ILC2-mediated pro-inflammatory effects still remains imprecise, particularly in the human system. Most extensively studied so far, the anti-inflammatory cytokine IL-10 was identified to also suppress the type-2 immune response induced by *ex vivo* stimulated ILC2s (80, 83). IL-10 is secreted by various immune cell types (e.g., macrophages, myeloid DCs, and specific Th cell subsets) (151) and can also be produced by all ILC subsets (80), suggesting mutual control. The potent induction of IL-10 was also described as an important effector mechanism underlying the immunomodulatory properties of IL-27 (152). However, murine studies revealed an additional direct inhibitory effect of IL-27 on ILC2s (50, 131), although the translation of these findings into the human system is still lacking. As another potentially regulatory cytokine, the suppressive function of TGF-β on the cytokine secretion of human ILC2s has been discussed, though controversially (80, 83), with the implication that its described inhibitory effects on ILC2s are dependent on experimental conditions, such as cytokine concentrations and stimulation protocols. Despite IL-10, IL-27 and potentially also TGF-β, type-I interferons and IFN-γ were able to efficiently regulate ILC2 activity in the murine ILC2s *in vitro* and *in vivo* (50, 84, 85, 131, 153). Although the translation of these data into the human system still remains incomplete, the impact of the type-I interferons IFN-α and IFN-β on the activation of regulatory pathways and the downregulation of type-2 cytokine production could successfully be confirmed for human ILC2s, respectively (84, 85).

Next to the active contribution of cytokines, lipid mediators represent another group of immuno-modulatory substances that regulate ILC2 activity, including the arachidonic acid metabolites prostaglandins, leukotriens, and lipoxins.

Most prominently, prostaglandin D_2_ (PGD_2_) has been shown to activate ILC2s via its G protein-coupled receptor CRTH2 (87, 88), which represents a classical marker for identifying human ILC2s (60). Large amounts of PGD_2_ are typically released from IgE cross-linked mast cells during an allergic reaction, resulting in the secretion of pro-inflammatory cytokines by ILC2s as well as the induction of IL-33R expression, further boosting the inflammatory response (87). A more recent study even described an auto- or paracrine stimulatory effect of ILC2-derived PGD_2_ (154). Given the increased pulmonary PGD_2_ levels observed in asthmatic and chronic rhinitis patients (155, 156), this might further explain the active contribution of ILC2s in allergic diseases.

In contrast to the activating properties of PGD_2_, PGI_2_ was assumed to restrict ILC2 effector functions. This was based on the *in vitro* finding that the PGI_2_ analog cicaprost reduced IL-2- and IL-33-induced type-2 cytokine production in human blood ILCs. The *in vivo* relevance of this finding was demonstrated in mice with allergen-induced lung inflammation, which displayed reduced pulmonary ILC2 counts after cicaprost treatment and a dependency on PGI_2_ receptor signaling (90). However, further proof is necessary to validate these initial findings. Furthermore, another study indicated an inhibitory effect of PGE_2_ on human blood and tonsilar ILC2s mediated via the E-type prostanoid receptors (EP) 2 and EP4. In the presence of PGE_2_, alarmin-induced secretion of IL-5 and IL-13, expression of GATA3 and CD25, and ILC2 proliferation turned out to be significantly decreased. EP2 and EP4 receptors might thus represent promising target structures for a potential therapeutic modulation of the overwhelmingly activated ILC2 axis in allergic diseases (91).

Following the detection of functional cysteinyl leukotriene receptor 1 (CysLTR1) expression on human blood ILC2s, the receptor ligands LTC_4_, LTD_4_, and LTE_4_ have been identified as additional activators of human ILC2s. In particular, LTE_4_ was described as a potent stimulator of ILC2 viability and effector cytokine secretion, with IgE cross-linked mast cells being one of its main producers *in vivo*. Regarding the complex multifactorial situation of tissue inflammation, the alarmins IL-25, IL-33, and TLSP and also PGD_2_ were found to amplify the LTE_4_-induced effector-cytokine secretion. The CysLTR1 antagonist montelukast, which is clinically approved, for instance, for asthma therapy, was able to inhibit this LTE_4_-induced ILC2 activation (89). Interestingly, PGD_2_ and the cysteinyl leukotriens LTC_4_, LTD_4_, and LTE_4_ not only activate ILC2s but also harbor chemotactic potential, driving the accumulation and thereby the numerical regulation of local ILC2s (for more details see the chapter Tissue-Specific Migration of ILCs During Adulthood) (87, 89).

Another class of lipid mediators, the lipoxins, are known for their pro-resolving function (157). In line with this, lipoxin A4 has been described to suppress cytokine-induced IL-13 release from human blood ILC2s via the ALX/FPR2 receptor (88).

In addition, the active metabolites of vitamin A and D were found to significantly influence the effector cytokine secretion of human blood ILC2s. While the vitamin A metabolite retinoic acid enhanced the secretion of IL-5 and IL-13 by activated ILC2s as well as the expression of α4β7, the vitamin D metabolite 1,25D exhibited suppressive functions (92).

In the last decade, intense research on human ILC2s has discovered a broad regulatory network mainly consisting of cytokines and lipid mediators controlling human ILC2 activity. If dysregulated, reduced or overwhelming ILC2 responses might lead to parasitic infections and chronic inflammation, respectively (129, 158). Serving as central activators or suppressors of ILC2 responses, the identified soluble mediators and their respective receptors might be of high therapeutic relevance in ILC2-driven diseases. Hence, the identification of further mechanisms regulating ILC2 activity in humans is of great clinical value. Results from murine studies suggest additional classes of potent ILC2 mediators, including hormones and neuropeptides, as well as exogenous agents, like bacterial products, that might serve as potential therapeutic targets. Dihydrotestosterone, a metabolite of the sex hormone testosterone, for instance, was suggested to restrict ILC2 differentiation via androgen receptor signaling, resulting in reduced lung ILC2 numbers in male compared to female mice, both in steady-state and upon allergen-induced lung inflammation (159, 160). This might potentially explain the increased prevalence of asthma in adult women compared to men (160). Moreover, with the identification of the inhibitory impact of β2-adrenergic receptor signaling on murine ILC2 proliferation and activity (161), a new interesting field of ILC2-neuronal cross-talk has been opened up. This was further expanded by the description of the neuropeptides neuromedin U and calcitonin gene-related peptide (CGRP) as efficient positive and negative regulators of murine ILC2s, respectively (162–165). Furthermore, exogenous mediators, including, for example, bacterial products upon infection (153), have been suggested to alter murine ILC2 activity. To serve as potential therapeutic targets, however, translation of these results into the human system and deeper research on the behavior of human ILC2s is mandatory.

Collectively, a plethora of soluble ILC2 regulators have already been identified. Their importance for ILC2 activation or inhibition, however, might vary depending on the tissue-specific phenotype and function of ILC2s (146, 147). A more detailed analysis of organ-specific ILC2 regulation will therefore help to evaluate the potential of ILC2 regulators as therapeutics targets in future.

##### ILC2-cell interactions

Whereas numerous soluble mediators have been identified that modulate the activity of human ILC2s, they can also be regulated by direct cell-cell interactions with other immune cells, endothelial cells, and stromal cells, in total providing a tight control network (Figure 1).

Originally known to mediate firm contact between circulating immune cells and the vascular endothelium and thereby initiating the homing process of lymphocytes into tissues, intercellular adhesion molecules, like ICAM-1 (intercellular adhesion molecule 1) and its integrin ligand LFA-1 (leukocyte function-associated molecule-1), can also provide stimulatory signals between immune cells. Interestingly, human blood ILC2s turned out to express both ICAM-1 and LFA-1, suggesting a potential interaction of ILC2s with each other. And indeed, ICAM-1–LFA-1-mediated contact of human ILC2s efficiently induced IL-5 and IL-13 secretion *in vitro*, which could be significantly diminished in the presence of ICAM-1 or LFA-1 blocking antibodies (93). Upon stimulation by IL-33, which is rapidly released by epithelial cells sensing stress signals *in vivo* (166), ICAM-1 expression was upregulated in human ILC2s (93), indicating the importance of this interaction for mounting efficient ILC2 responses. Using a mouse model of IL-33-induced lung inflammation, the pathophysiological *in vivo* relevance of this interaction could be strengthened: blocking the CD11a subunit of the ligand LFA-1 resulted in decreased signs of lung inflammation in immunodeficient Rag1^−/−^ mice (93). Experiments with murine ILC2s further elucidated GATA3 and subsequent ERK signaling as a central downstream mechanism of ICAM-1–LFA-1-mediated ILC2 activation (93). ICAM-1-expressing endothelial cells represent further potential interaction partners of LFA-1^+^ ILC2s, and data from the murine system suggested that the LFA-1 subunit β2 drove the migration of blood ILC2s into the inflamed lung tissue (167). Having shown that human ILC2s express functional LFA-1 (93), this might also be relevant in the human ILC2 lung homing process.

Furthermore, co-stimulatory signals have been described to markedly contribute to ILC2 activation, including molecules of the TNF receptor as well as the B7-CD28 superfamilies. For the TNF receptor superfamily member GITR (glucocorticoid-induced TNFR-related protein) and its ligand GITR-L, for instance, a substantial role in ILC2 activation has been indicated (94). Whereas, GITR-L is primarily expressed by APCs and endothelial cells (168), murine and human ILC2s expressed functional GITR that, upon binding to GITR-L or respective agonists, induced ILC2 proliferation as well as upregulation of effector cytokine transcripts (94). Based on murine data, the stimulatory effect of GITR engagement was based on its synergistic effect with IL-33 on the induction of IL-9 expression, which, in turn, upregulated IL-5 and IL-13 in an autocrine, STAT5-dependent fashion (94). In line with this, the interaction of GITR and its ligand appeared to be important for the pulmonary development of allergic inflammation (94). Moreover, human blood and nasal polyp ILC2s were found to express RANK (receptor activator of nuclear factor κ B), another member of the TNF receptor superfamily, which was suggested to be of biological importance in chronic rhinosinusitis patients with nasal polyps. In this context, the ligand RANK-L was mainly expressed by CD45^+^ immune cells, including Th2 cells, and its levels were significantly increased in nasal polyps. Successful RANK–RANK-L engagement stimulated human ILC2s to secrete enhanced IL-5 and IL-13 levels via NFκB signaling and acted in synergy with TSLP (95). Given the stimulatory effects of TNF receptor superfamily members expressed by ILC2s on the induction of type-2 airway inflammation, they might present promising new therapeutic targets in the future. The B7-CD28 superfamily member ICOS and its ligand ICOS-L, which have been described extensively as co-stimulatory molecules in the antigen-specific interaction between Th cells and APCs (169, 170), have also been described as potent auto-stimulatory triggers for the antigen-independent activation of ILC2s. Both functional ICOS and ICOS-L are expressed by human blood ILC2s, where their cell contact-dependent interaction induced a significantly increased production of IL-5 and IL-13 by *in vitro* stimulated ILC2s. In line with this, experimental *in vitro* and *in vivo* blockade of ICOS signaling markedly inhibited the pro-inflammatory properties of human ILC2s, resulting in reduced airway inflammation in a humanized mouse model of IL-33-induced airway hyperreactivity (96). Accordingly, increased numbers of ICOS^+^ ILC2s were detected in the BAL of patients with idiopathic pulmonary fibrosis compared to control subjects (37), further indicating a relevant function of ICOS signaling in ILC2s in the diseased lung. Surprisingly, another study demonstrated that the inhibitory effect of induced Tregs on human ILC2 activity could be blocked efficiently by ICOS-L neutralizing antibodies *in vitro* and *in vivo*. The authors thus postulated a direct interaction between ICOS-L^+^ ILC2s and ICOS^+^ induced Tregs that efficiently suppressed ILC2 effector functions and might therefore act as crucial mediators for the resolution of lung inflammation (97). Taken together, ICOS-L signaling might have contrary roles in human ILC2s depending on the ICOS-expressing interaction partner, which might potentially compete for contact with ICOS-L^+^ ILC2s. (171). Moreover, data from murine experiments suggest that ICOS-L-expressing DCs might serve as an additional interaction partner for ICOS^+^ ILC2s and thus support allergic lung inflammation (172).

Besides their essential molecular involvement in the process of antigen presentation by professional APCs, MHCII molecules have also been shown to be expressed by non-classical APCs, including human ILC2s (173). Oliphant and colleagues detected the expression of both the MHCII molecule HLA-DR and the co-stimulatory CD28 ligands CD80 and CD86 on the surface of human blood ILC2s, allowing the efficient processing and presentation of antigens to Th cells *in vitro* (34). The functional relevance of this observation was further analyzed in the murine system, showing a reciprocal, MHCII- and CD80/CD86-dependent crosstalk between antigen-presenting ILC2s and Th cells in the presence of the cognate antigen that was important for the successful expulsion of *Nippostrongulus brasiliensis* infections. This interaction not only led to the activation of antigen-specific T cells but also triggered ILC2 expansion and IL-13 production via T cell-derived IL-2. ILC2 stimulation was therefore suggested to be initiated by the epithelial cell-derived alarmins IL-25 and IL-33 but to be maintained by IL-2 secreted by T cells upon MHCII–TCR interaction with ILC2s (34).

Originally, the natural cytotoxicity receptor NKp30 was identified as an activating receptor on NK cells mediating the elimination of tumor and virus-infected cells (174). However, it was also found to be highly expressed on blood and *ex vivo* cultured human ILC2s. Upon interaction with the plate- or membrane-bound NKp30 ligand B7-H6, NKp30^+^ ILC2s were stimulated to secrete increasing amounts of IL-13, while the mRNA expression of important activating receptors, including ST2, CRTH2, and IL-17RB, was downregulated. This was suggested to serve as a negative feedback mechanism regulating the activation status of pro-inflammatory ILC2s. Besides tumor cells, B7-H6 could also be detected on the basal epidermis of healthy individuals and even in the suprabasal epidermis layers of atopic dermatitis patients, implying a role of NKp30–B7-H6 signaling in the activation of human skin ILC2s during chronic inflammation (98). B7-H6 expression was additionally found in some tumor samples as well as adjacent normal lung tissue (175), suggesting a potential role in the activation of pulmonary ILC2s, as well. Whether the NKp30-mediated ILC2 stimulation can also be induced by other NKp30 ligands like BAT3 or BAG6 still needs to be clarified.

While a variety of cell-cell contact-dependent ILC2 activators have been identified, there is considerably less understanding of interactions limiting ILC2-mediated inflammation.

Being known as a cell adhesion molecule that provides intercellular junctions between epithelial cells and thereby guarantees a stable barrier as the first line of physical immune defense, E cadherin (epithelial cadherin) can also interact with KLRG1 (killer cell lectin-like receptor G1)-expressing immune cells (176, 177). Interestingly, upregulation of KLRG1 surface expression was observed in human skin ILC2s under inflammatory *in vitro* and *in vivo* conditions. On a functional level, binding of KLRG1 to its ligand E cadherin resulted in significantly decreased proliferation and effector cytokine expression of human ILC2s *in vitro* (54). In the pathological context of atopic dermatitis and asthma, this suppressive mechanism was suggested to be impaired based on reduced local expression of E cadherin in both diseases (54, 178), which finally results in ILC2-driven chronic inflammation. Due to the rather broad expression profile of the adhesion protein E cadherin in different epithelial organs (179–181), the suggested KLRG1-dependent mechanisms might represent an important activation-induced negative feedback loop allowing the termination of local ILC2 responses at different sites of the human body.

The controlled resolution of ILC2-driven immune reactions might further be supported by the checkpoint inhibitor PD-1 (programmed cell death protein 1), which was co-expressed by a relevant subset of KLRG1^+^ human blood ILC2s. Experimental blockade of PD-1 signaling in human ILC2s significantly enhanced their proliferation and IL-33-induced cytokine production via the STAT5 pathway. Together with the *in vivo* finding that functional PD-1 signaling hindered murine ILC2s to efficiently clear *Nippostrongylus brasiliensis* infections, these results implied a role for PD-1 as an important checkpoint inhibitor regulating activated ILC2s. Although the interaction partner of PD-1^+^ ILC2s has not yet been analyzed in humans, the PD-1 ligands PD-L1 and PD-L2 are classically induced in various immune cell types (182). Murine data even demonstrated that ILC2s themselves can express PD-L1, which was upregulated upon type-2 inflammation. Unexpectedly, PD-L1^+^ ILC2s stimulated PD-1-expressing CD4^+^ T cells rather than suppressing them (33), demanding deeper research into the PD-1 and PD-L1 functions in human ILC2s.

Collectively, our current knowledge on the regulation of human ILC2s indicates the existence of a tight network involving numerous control mechanisms but also offering many potential cellular and molecular targets for dysregulation.

#### Local Regulation of Human Helper ILC3s

By secreting IL-22 and IL-17, helper ILC3s are crucial for preserving the barrier integrity of mucous epithelia and thereby protecting the host against invading pathogens. However, when dysregulated, the host-protective functions of ILC3s can transform into detrimental immune activation, finally leading to chronic inflammation (183–185). So far, ILC3 research has primarily focused on their function in the intestine, where IL-22-expressing ILC3s are present even under steady-state conditions, while only very low numbers of IL-17-producing ILC3s could be detected in the non-inflamed human gut (6).

Classically known from the maintenance of Th17 cells in the adaptive immune system (186), the cytokines IL-23 and IL-1β also represent prototypical inducers of IL-22 secretion by human ILC3s (30, 52, 142, 187) and are mainly released by DCs and epithelial cells upon tissue inflammation (6). Thus, IL-23 and IL-1β serve as potent mediators that translate the intestinal penetration of commensal and pathogenic bacteria into the induction of a tissue-protective immune response initiated by ILC3-derived IL-22 via CD11c^+^ myeloid DCs. Indeed, human intestinal ILC3s that had been in contact with fecal bacteria in the intestine were characterized by increased IL-22 production *ex vivo* compared to those derived from tissue sites without fecal bacteria exposure (30). Interestingly, this indirect stimulation of human ILC3s by bacteria was more pronounced in intestinal ILC3s than in tonsillar ILC3s (188), suggesting a tissue-specific regulation of this phenomenon. Independent of accessory cell mediators, bacterial products can also directly induce the proliferation and cytokine production of ILC3s via the activation of Toll-like receptor (TLR) signaling, as shown for NFκB-dependent TLR2 activation in tonsillar human LTi ILC3s in the presence of IL-2 (103). Moreover, products of the bacterial tryptophan metabolism are suggested to directly stimulate ILC3s via binding to the aryl hydrocarbon receptor (AHR), which was shown to be expressed on human ILC3s (104, 105). The functional relevance of AHR signaling on ILC3s was later demonstrated in mice in the context of resolution of *Citrobacter rodentium* infection (189). In contrast, other bacterial products inhibit ILC3 activity, likely to delay epithelial repair and favor their own dissemination. A candidate for this is the *Bacillus anthracis* toxin, which could be shown to suppress IL-22 production by IL-23-stimulated human ILCs *in vitro* via MAPK signaling disruption (106).

Under *in vitro* conditions, ILC3 proliferation and IL-22 secretion could also be induced by the combined effect of the survival factor IL-15 and the pro-inflammatory cytokine IL-18. The stimulatory effect of IL-18 was mediated via ligation of the IL-18Rα and IL-18Rβ subunits on the surface of tonsillar human ILC3s, resulting in functional signaling of the heterodimeric IL-18 receptor, subsequent NFκB activation and finally the transcription of the *IL22* gene (100). *In vivo*, IL-18 secretion could be detected in CD11c^+^ DCs located in direct proximity to ILC3s in human tonsils (100), enabling paracrine ILC3 stimulation. Moreover, increased IL-18 levels (190) together with the enhanced IL-22 secretion observed in ileal ILCs from CD patients (30) indicate a significant role of IL-18 stimulated ILC3s in the pathological context of CD.

Data acquired in a murine model of spontaneous colitis and *in vitro* analyses of human LPMCs additionally demonstrated a certain stimulatory function of the pro-inflammatory cytokine IL-6 on the ILC3-mediated cytokine secretion in the gut (101). Colon explant cultures of IBD and control subjects further detected a subgroup of IBD patients with high IL-6 production compared to controls (101), implying that IL-6 might be, at least partly, responsible for the increase in IL-17-expressing mucosal ILCs observed in a subgroup of CD patients (52).

In addition to its functional impact on ILC2s (28), the DR3 ligand TL1A also acts as a co-stimulatory trigger for the IL-1β- and IL-23-induced cytokine production and proliferation of human ILC3s, as shown in both stimulated intestinal and *in vitro* differentiated human ILC3 cultures (30, 102, 191). Mechanistically, TL1A was suggested to induce the expression of the IL-2 receptor subunit CD25 on TL1A-stimulated ILC3s and thus to prime ILC3s for acquiring proliferative signals via IL-2 (192). The idea of a functional DR3-TL1A interaction on human ILC3s was further strengthened by the finding that human ILC3s expressed DR3 transcripts even under resting conditions (192). Under pathophysiological conditions, microbial-sensing mononuclear phagocytes appeared to be an important source of TL1A. They were thus able to initiate an anti-microbial, tissue-restoring immune response (30) and should be taken into account, especially in the context of IBD. In line with this, inflammatory intestinal tissue sites of IBD patients were characterized by increased levels of IL-22, likely derived from ILC3s (30). In parallel, intestinal inflammation in IBD patients is associated with an accumulation of IL-17^+^ ILC3s in the ileum and colon and an increased capacity of IL-23 to trigger the expression of IL-17A in gut-derived ILC3s (6, 52).

Besides the here described involvement of cytokines (Table 1), mucosal immune cells, and bacteria in the ILC3-activating machinery, several other factors have been suggested to be crucial promotors of local ILC3 accumulation and function in humans, such as neurotransmitters, vitamin metabolites, and even lifestyle (e.g., obesity and cigarette smoking) (107, 108, 193, 194). In the case of neurotransmitters, vagus-derived acetylcholin was described to stimulate the PCTR1 pathway in both murine and human ILC3s, favoring the resolution of inflammation (107). Moreover, the enteric neuron-derived vasoactive intestinal peptide (VIP) was shown, at least in mice, to modulate ILC3 activity upon food intake, though with controversial effects (195, 196). Ingested as a food component or directly synthesized in sun-exposed skin, the active metabolite of vitamin D, 1,25D, was additionally described to alter the transcriptional profile of human ILC3s, skewing them toward the IL-1β pathway while downregulating IL-23R signaling at the same time. In IBD, where vitamin D deficiency has been reported to be a risk factor, the observed beneficial effects of vitamin D substitution (197) might thus mechanistically include the inhibition of IL-23- and IL-17A-secretion by ILC3s (108). In general, only little is clearly known about the mechanisms negatively regulating human ILC3 proliferation and their activity so far. The first hints of potential ILC3 cytokine inhibitors were acquired from *in vitro* stimulated human tonsillar ILC3s only and demonstrated the suppressive effect of recombinant human IFN-α and IFN-γ on ILC3 numbers (100). Future research should therefore intensify its work on the identification of inhibitors regulating ILC3 activity in order to potentially pave the way for novel therapeutic strategies in inflammatory diseases characterized by an overwhelming ILC3 activity, like IBD.

### ILC Plasticity and Tissue Differentiation

Since a markedly altered local ILC composition has been described in inflammatory diseases (75, 183, 198–200), it is important to understand the underlying mechanisms as well as the pathological relevance of this observation. Changes in local cell numbers can be explained by cell death, local proliferation, intercompartmental redistribution, or directed recruitment of existing ILC fractions from distal sites. Moreover, the differentiation of tissue-resident ILC precursors and the transdifferentiation of mature ILCs (Figure 2) can also contribute to altered ILC numbers in inflammatory tissue sites (Figure 1), allowing adaption to local requirements without recruiting additional cells (201). While initial studies identified three helper ILC subsets, a more complex diversity has now been described (10, 104, 202), including intermediates between distinct mature subgroups and ex-ILCs derived from the transdifferentiation of one ILC subgroup into another (202).

**Figure 2:** (Trans-) Differentiation of human ILCs in mucosal tissues. To adapt the local pool of tissue-resident ILCs, mature ILCs can differentiate from local precursors or transdifferentiate into other ILC subsets. This shift in local ILC subgroups is mediated by the local cytokine environment and can be observed in various fibro-inflammatory diseases affecting the lung and gut. CD and severe COPD, for instance, are characterized by an ILC1-dominated immune response. In line with this, human ILC1s can be induced from c-Kit^+^NKp44^−^ ILC precursors as well as from mature ILC2s and ILC3s in these pathologies; this is mainly regulated by IL-12. In contrast, in chronic rhinosinusitis with nasal polyps (CRwNP), ILC2s rather than ILC1s represent important effector cells triggering the immune response. Accordingly, ILC2 plasticity can be suppressed by IL-4 and vitamin D3, hampering the acquisition of ILC1- or ILC3-like characteristics to preserve type-2 immunity. Nevertheless, retinoic acid can trigger ILCreg formation from mature ILC2s, likely representing a negative feedback mechanism to control ILC2 responses. Though characterized by nasal polyps as well, cystic fibrosis patients (CFwNP) display an ILC3-driven phenotype in upper airways that can be induced by TGF-β-driven transdifferentiation of ILC2s into ILC3s. Potentially, ILC1s might also represent a source of mature ILC3s, as shown *in vitro* in response to IL-23, TGF-β, and retinoic acid. Whether further ILC plasticity exists in humans needs to be targeted in future studies.

#### ILC3 ↔ ILC1 Plasticity

ILC plasticity seems to be particularly interesting in pathologies characterized by the increase of one ILC subgroup at the expense of another. This was observed, for instance, in CD patients, who are characterized by having enhanced ILC1 frequencies in inflamed intestinal tissue with a simultaneous decrease in the NKp44^+^ ILC3 population compared to non-inflamed control tissue (15). Searching for a functional link between these associated phenomena, it was important to learn that the type-1 cytokine IL-12 not only represents a potent ILC1 activator (44) but also serves as a key inducer of ILC3-to-ILC1 transdifferentiation. *In vitro* experiments with human tonsillar and fetal gut ILC3s confirmed the plasticity of mature ILC3s, differentiating into IFN-γ-producing ILC1s upon IL-2 and IL-12 stimulation with or without the addition of IL-1β (15, 201, 203). Moreover, TGF-β was also suggested to induce T-bet expression in stimulated human ILC3s (202). *Ex vivo* analyses of human ileal LPMCs revealed the existence of ILC subgroups in the transition phase that share both ILC3 and ILC1 characteristics, thus hinting at a biological relevance of the ILC3-to-ILC1-shift even in the complex *in vivo* situation (202). This was further proven in a humanized mouse model: after adoptive transfer of *ex vivo* expanded IL-22-secreting human ILC3s, an organ- and time-dependent switch to IFN-γ secretion was observed (202). For transition, the transcription factors Aiolos and Ikaros were suggested to shut down the transcription of ILC3 signature genes, thereby allowing the induction of an ILC1-like phenotype and function (202, 203).

Conversely, the combined effects of IL-2, IL-23, and IL-1β induced the phenotype and function of mature ILC3s in former human ILC1s, including RORC expression and IL-22 secretion, which could be further triggered by the vitamin A metabolite retinoic acid. Indeed, the intravenous transfer of human ILC1s into a humanized mouse model resulted in the appearance of human NKp44^+^ ILC3s in the gut of recipient animals, further proving the *in vivo* validity of the ILC1-to-ILC3 switch even under non-inflammatory conditions (201). In the pulmonary mucosal tissue, the clinical significance of the ILC3-to-ILC1 shift was described in the tumor context in patients with pulmonary squamous cell carcinoma. Induced by IL-23-secreting tumor cells, human lung ILC1s gave rise to functional ILC3s and thereby supported IL-17-mediated tumor growth. This was, in particular, reflected by the finding that high ILC3 numbers and IL-23 and IL-17 levels turned out to significantly correlate with decreased patient survival (204). An even higher level of flexibility in the ILC1/ILC3 ratio is achieved by the availability of local immature human ILCs (c-Kit^+^NKp44^−^), which can undergo differentiation toward either functional ILC1s or NKp44^+^ILC3s in the presence of IL-2 and IL-12 or IL-2, IL-23, and IL-1β, respectively (15).

#### ILC2 ↔ ILC1 Plasticity

Another ILC1-dominated disease, COPD, is characterized by enhanced ILC1 frequencies at the cost of ILC2s in the peripheral blood and also the inflamed lung tissue (55, 200). Since the number of total ILCs was unaffected by the IL-12-enriched inflammation in COPD patients (200), the transdifferentiation of mature ILC2s into functional ILC1s might explain this inverse correlation of ILC1 and ILC2 frequencies, pointing to the ILC1-inducing cytokine IL-12 as a candidate mediator. And indeed, *in vitro* stimulated human ILC2s lost their type-2 characteristics in the presence of IL-12 and acquired the phenotype and function of ILC1s instead (55, 200). Interestingly, IL-1β was found to further support the ILC2-to-ILC1 shift by priming ILC2s for optimal response to IL-12 (82). In particular, a subset of IL-13^+^ human ILC2s turned out to co-express IFN-γ in response to strong IL-12 signaling (205). Accordingly, ILC2s derived from IL-12Rβ1-deficient patients with mendelian susceptibility to mycobacterial disease were unable to exhibit ILC2-to-ILC1 plasticity while intestinal samples from CD patients harbored transdifferentiated IL-13^+^IFN-γ^+^ ex-ILC2s (205). The functional relevance of the described ILC2-to-ILC1 switch for the clinical course of inflammatory pathologies was further confirmed by showing a positive correlation between increased ILC1/ILC2 proportions in COPD patients and augmented symptoms of respiratory disease (200). Chronic exposure to cigarette smoke and respiratory tract infections, known to be strongly associated with the occurrence of COPD, might further trigger this conversion (200). Surprisingly, the classical type-2 cytokine IL-33 was able to enhance the IL-12-induced IFN-γ production in human ex-ILC2s, indicating a dual, context-dependent role of IL-33 (200). In contrast, IL-4 acted as a classical type-2 cytokine and could reverse human ex-ILC2s into functional ILC2s again *in vitro* and might thus be able to support the maintenance of an ILC2 predominance in mucosal tissues, as observed in patients suffering from chronic rhinosinusitis with nasal polyps. An increased proportion of ILC2s was detected in the turbinate tissue of these patients, while the local frequencies of ILC1s and ILC3s were diminished. This observation might be partly explained by the co-localization of ILC2s with IL-4-secreting eosinophils and the capacity of IL-4 to stabilize the phenotype and function of ILC2s (55). However, besides the described capacity of IL-4 to re-convert ex-ILC2s to their initial ILC2 phenotype, there have been no reports describing milieu-dependent transdifferentiation of human ILC2s from bona fide ILC1s or ILC3s (55). Also, in the clinical context of chronic rhinosinusitis, nasal polyps of affected patients showed an increased frequency of ILCregs (206). Similar to Tregs, their counterparts in the adaptive immune system, ILCregs possess a regulatory capacity exerted via the secretion of the immunosuppressive cytokine IL-10 (22). Interestingly, ILC2-to-ILCreg transdifferentiation seemed to appear in the presence of retinoic acid and resulted in marked IL-10 secretion by former human ILC2s (206).

#### ILC2 ↔ ILC3 Plasticity

Unlike the type-2 signature dominating the immune response in nasal polyps of patients with chronic rhinosinusitis, cystic fibrosis patients with nasal polyps exhibited a substantially increased frequency of NKp44^−^ ILC3s compared to chronic rhinosinusitis patients, even though nasal polyps in the two diseases share morphological and clinical characteristics (72). Based on *in vitro* data showing the transdifferentiation of human ILC2s into ILC3-like cells in the presence of TGF-β, an ILC2-derived IL-17-secreting ILC3-like subtype was suggested to be responsible for this observation (72, 207). Consistently, increased TGF-β levels have been described in nasal polyps of cystic fibrosis patients (72). In this context, epithelial cell-released TGF-β was suggested to induce SMAD2/3 phosphorylation in nasal human ILC2s and thereby initiate their transdifferentiation into IL-17A-secreting ILC3s. In turn, ILC-derived IL-17A can recruit neutrophils and thus further promote inflammation (72). A similar switch of the c-Kit^−^ ILC2 subgroup was observed in psoriatic skin lesions, identifying mutual control of GATA3 and RORγt expression as an important control center deciding the fate of ILC2s (207). Through cell culture experiments, IL-4 and vitamin D3 could be revealed as antagonists of this ILC plasticity, suppressing the TGF-β-initiated subtype switch (72, 207). The biological impact of this ILC2-to-ILC3 conversion, however, is restricted to the skin (207) and upper airways (72) so far, and whether this also applies to the lower airways and other organs needs to be addressed in future studies (202). In addition, it is still insufficiently clarified whether ILC2s can fully convert into ILC3s or whether they might keep certain ILC2 characteristics as ILC3-like cells (207). This also raises the question of whether multistep ILC plasticity is possible or whether there are specialized subsets of ILC1s, ILC2s, and ILC3s that can only adapt defined characteristics of another subgroup.

Although experimental proof of ILC3-to-ILC2 plasticity in humans is lacking to date, it was interesting to note the identification of lin^−^CD117^+^CD127^+^ LTi-like cells as an intermediate subset between LTi ILC3s and functional ILC2s. Assuming that there was no contamination of this cell population with mature ILC2s, simultaneous production of the type-3 cytokine IL-22 and the type-2 cytokines IL-5 and IL-13 has been demonstrated in response to PMA, ionomycin, and brefeldin A in expanded human CD127^+^ LTi-like cells. Moreover, clonal expansion of LTi-like cells revealed heterogeneous effector cytokine profiles of analyzed clones, which were skewed either to the type-3 or the type-1 side but showed comparable RORC and GATA3 levels (103). Thus, LTi-like cells might represent an intermediate or precursor ILC subset. Stimulation with IL-2 or IL-15 and the TLR2 ligand Pam3 increased the IL-13 and IL-22 secretion by human LTi-like cells *in vitro*, while only the minority of cells were IL-22^+^ (103), indicating that bacterial products might directly activate LTi-like cells and, in combination with further stimuli, might decide the fate of this intermediate ILC subset. Further research, however, is necessary to confirm the direct link between the described LTi-like cells and the transdifferentiation of ILC3s into ILC2s. In another study, KLRG1^+^ ILCs were additionally suggested as intermediate cells biased toward the ILC2 lineage but with the potential to differentiate into IFN-γ- and IL-22-producing ILCs upon stimulation with IL-1β and IL-23 (208). Similarly, NKp46^+^ ILCs were postulated to represent ILC3 precursors but with the ability to generate ILC1- and NK cell-like ILCs upon IL-12 treatment (208).

Collectively, human ILCs have been described as highly plastic cells (Figure 2). Indeed, many key cytokines regulating ILC activity have been demonstrated not only to control the proliferation and effector cytokine secretion of a distinct ILC subgroup but also to mediate the transdifferentiation of ILCs. Thus, dependent on the environmental stimuli, the plasticity of mature ILCs and the differentiation of local ILC precursors enable a rapid and reversible adaption of the ILC pool to local requirements and subsequent modulation of the innate immune response.

### Tissue-Specific Migration of ILCs During Adulthood

In humans, relatively small but distinct populations of ILC precursors and even mature ILCs are present in the peripheral blood stream during child- and adulthood (26, 51, 80, 208). Yet, their functional role in the circulation itself or on local immune responses has not been fully elucidated. Since disease-associated tissue inflammation, as observed for instance in asthma, is not only reflected in an adapted local ILC pool but also in altered ILC frequencies in the peripheral blood (31, 64), a biological impact of circulating blood ILCs on systemic or local immune responses is strongly suggested. Functional data acquired in parabiotic mouse models initially argued against this, establishing a paradigm of tissue-resident ILCs that are, at least in the murine organism, incapable of homing from the blood stream to the inflamed tissue site (49, 50). Nowadays, the concept of a strict tissue residency of ILCs has become outdated, superseded by the idea of a rather time- and context-dependent homing capacity of blood ILCs (209) as a response to steady-state losses or under inflammatory conditions. Even in the model of parabiotic mice, a small but significant homing of blood ILC2s into tissues could be overserved upon chronic inflammation (49). In line with this, a recent study described an infection- and inflammation-triggered interorgan migration of gut-resident ILC2s via S1P-mediated chemotaxis in mice. In particular, intestinal inflammatory ILC2s were identified to be a migratory ILC subset that played a crucial role in clearing helminth infections and restoring epithelial tissue integrity, not only in the gut but also in the distant lung tissue (35). Regarding the translatability of the concept of trafficking ILCs into the human system, expression of functional S1P receptors was also proven in human tonsillar ILC1s, ILC2s, and ILC3s. *In vitro*-performed chemotaxis assays further confirmed active migration of human ILC1s and ILC3s in response to S1P analogs with a prominent role of S1PR1, while ILC2s were not analyzed in this context. *In vivo* therapy of patients with relapsing-remitting multiple sclerosis with the S1P agonist fingolimod resulted in an impressive reduction of all ILC subgroups in the peripheral blood, suggesting S1P-dependent trafficking of blood ILCs into lymph nodes in the human *in vivo* situation, too (210). In a completely different clinical setting, partial repopulation of ILC niches with ILCs after myeloablation was shown to take place postnatally in patients with severe combined immunodeficiency after hematopoietic stem cell transplantation (26). These results indicated the migration of donor-derived ILCs or their precursors to replenish blood and tissue ILCs even after birth and fit very well with the recently postulated model of tissue-specific “ILC-poiesis.” With the identification of uni- and multipotent CD117^+^ ILC precursors in peripheral human blood, milieu-driven recruitment and local maturation of blood-derived ILC precursors has been suggested to replenish and adapt the pool of tissue-resident mature ILCs (51). As well as these circulating CD117^+^ ILC precursors, mature ILCs also exist in the blood stream (26, 60, 80) and show a characteristic surface expression profile of chemokine receptors and integrins, which are generally known as key regulators of tissue-specific homing processes (211). Circulating ILC1s expressed varying levels of CCR4 and CCR6 and were mainly characterized by high frequencies of CCR7^+^, CXCR3^+^, and α4β7^+^ cells but lower percentages of CCR5^+^, CCR9^+^, and CXCR6^+^ ILC1s (53, 212). In contrast, the vast majority of human blood ILC2s expressed CCR4, CCR6, and the integrins α4, αL, β1, and β2 and additionally displayed distinct but smaller subsets of CCR9^+^ and β7 integrin^+^ cells (53, 167, 212). Only rare ILC2 subsets expressed CCR5, CCR7, and CCR10, while CXCR3, CXCR5, and CXCR6 were almost absent on blood ILC2s (53, 212). While expressing CCR4 and CCR6 in varying levels as well (53), human blood ILC3s differed from other helper ILCs by the expression of CCR10 and cutaneous lymphocyte antigen (CLA) (212). However, they also showed small fractions that stained positive for CXCR3, CCR7, and α4β7 integrin (53, 212). In adaptive immune cells, several of those chemokine receptors have been inferred to drive organ-specific homing pathways that might be translatable to ILCs as innate counterparts of Th cells. CCR7, for example, is known to drive homing to lymphoid tissues, while α4β7 integrin and CCR9 are specific for intestinal migration (213). CLA was suggested to promote homing processes to the skin (214). Whether this concept actually applies to human blood ILCs, however, needs further validation on a functional level. As a first step, the general homing capacity of human blood ILCs could be demonstrated in humanized mouse models: intravenously injected human ILCs could later be detected in various organs as tissue-resident cells (55, 201). Moreover, *in vitro* chemotaxis assays further elucidated specific ligand-receptor interactions regulating the controlled attraction of ILCs. Most prominently, the PGD_2_ receptor CRTH2 not only serves as phenotypical hallmark and activating receptor on ILC2s but could also promote directed *in vitro* migration of ILC2s toward PGD_2_ (87, 215, 216). Activated, IgE cross-linked mast cells were detected to be a major source of PGD_2_, suggesting a relevant role of the CRTH2–PGD_2_ interaction for mast cell-induced ILC2 recruitment upon allergic inflammation (87). In line with the accumulation of ILC2s in asthmatic lung tissue (31), ILC2s derived from asthmatic patients displayed enhanced migratory potential toward PGD_2_ compared to ILC2s from healthy subjects (216). The *in vivo* relevance of this CRTH2-driven ILC2 migration was underlined in mice confirming efficient PGD_2_-mediated accumulation of murine ILC2s in the lung and the importance of CRTH2 for efficiently mounting an anti-helminth lung inflammation (217). Likewise, the leukotriens LTE_4_, LTD_4_, and LTC_4_ also displayed chemotactic potential on human blood ILC2s, with LTE_4_ being the most potent chemotactic trigger when tested *in vitro* (89). Though less potent than PGD_2_ or LTE_4_ (87, 89), IL-33 could also trigger *in vitro* ILC2 migration (54, 87, 215). In contrast, other members of the ILC2 core activating unit, including IL-25 and TSLP, only showed a minimal chemotactic potential or were effective only at high concentrations, respectively (54, 87). Furthermore, TGF-β and the chemokine CCL8 could also attract human ILC2s in transmigration assays (215), which might be of functional relevance, as an accumulation of ILC2s could be detected in TGF-β-enriched asthmatic airways (218), and IL-33-induced lung inflammation in mice was associated with increased levels of peribronchial CCL8 (215). In tuberculosis-associated lung pathology, a reverse correlation of all ILC subsets has been observed with decreased frequencies in the peripheral blood, but an accumulation of these cells in the affected lung tissue, which was suggested to result from CXCL13–CXCR5-driven ILC lung homing. Thereby, migrated ILC3s were proposed to have a beneficial role against *Mycobacterium tuberculosis* in particular (69).

During the controlled process of immune cell homing, chemokine receptor-mediated signaling is of crucial importance for the activation of integrins expressed by rolling blood cells. Activated integrins mediate the actual adhesion of circulating immune cells to the endothelium (211). Phenotypically, a proportion of human blood and tissue ILC2s has been described to express the integrin subunits α4, αL, β1, and β2 (167). So far, the contribution of αLβ2 rather than α4 and β1 to the ILC2 lung homing process, however, has been functionally proven only in the murine system (167). In the context of gut immune homeostasis, intestinal DCs within mesenteric lymph nodes are specialized for metabolizing dietary vitamin A toward all-trans retinoic acid, which is known to induce membrane expression of α4β7 in CD4^+^ T cells and thereby imprints T cells for gut homing (219, 220). Thus, it was interesting to observe a similar increase in α4β7 expression on the surface of human blood-derived ILCs after *ex vivo* exposure to retinoic acid. In synergy with IL-2, retinoic acid successfully induced upregulation of α4 and β7 expression in ILC1s, ILC2s, and ILC3s and, in addition, also promoted a significant increase of β1 integrin levels in all three ILC subgroups (92). In contrast to the indicated capacity of retinoic acid to facilitate gut homing of ILCs via binding to the typical intestinal adhesion molecules MadCAM-1 and VCAM-1, vitamin D seems to counteract this effect. The retinoic acid-induced increase in surface expression of α4β7 integrins could be significantly inhibited by the vitamin D metabolite 1,25D in a dose-dependent manner (92).

Besides the influence of chemokines and integrins, the migratory behavior of ILCs might also be modulated by extracellular matrix proteins. In particular, type-I collagen was found to trigger changes in the cytoskeleton of human ILC2s, resulting in increased agility *in vitro*. Type-2 meditated inflammatory diseases of the lung might therefore be amplified by locally recruited and retained ILC2s upon pulmonary tissue remodeling (215).

Apart from the controversial discussion about the tissue residency or systemic mobility of human ILCs, they are assumed to be motile within tissues with a tightly controlled intra-organ localization and spatial distribution (215). But since functional data on human ILCs have been acquired in transmigration assays only, information on chemokines mediating inter- and/or intra-organ migration of ILCs is still lacking. Thus, based on the expression pattern of chemotactic mediators and their receptors, for now, it can only be speculated that, for example, CCR6-driven ILC2 migration might be particularly important for attracting ILC2s from the blood circulation to the tissue, since CCR6 expression is downregulated once ILC2s reside in the lung (221). In contrast, surface expression of integrin αE (CD103), and potentially also CXCR6, seems to predispose human NKp44^+^ ILC1s for intraepithelial accumulation (44). Interestingly, cell culture experiments indicated that the epithelium itself is able to control the maintenance of integrin αE expression on intraepithelial ILC1s via the release of TGF-β (44). Regarding the intra-organ distribution of ILC3s, the transmembrane chemotactic receptor GPR183 and its ligand 7a,25-dihydroxycholesterol were suggested to play a key role in the organization and localization of ILC3s within mesenteric lymph nodes, which might also be relevant in human GPR183-expressing ILC3s (222).

An augmented occurrence of highly organized ectopic lymphoid aggregates in, for instance, gut, lung, or liver tissue represents a frequently described feature of chronic inflammatory diseases like IBD, COPD, or rheumatoid arthritis, respectively (223). As LTi ILC3s crucially contribute to the formation of ectopic lymphoid aggregates via the secretion of lymphotoxin, IL-17A, and IL-22 (223), it was interesting to find a significantly increased number of neuropilin-1 (NRP1)-positive LTi cells in pulmonary tissue of COPD patients (224). Indeed, the adhesion molecule NRP1 turned out to represent a characteristic marker of human LTi ILC3, which impacts their chemotactic behavior functionally. *In vitro* analyses indicated that the chemoattractant vascular endothelial growth factor A (VEGF-A) was able to induce migration of LTi cells via engagement of NRP1 in complex with VEGFR2 (224). Together with a well-described upregulation of VEGF expression under chronic inflammatory conditions (225, 226), these findings strongly imply that the VEGF-A—NRP1-dependent recruitment of LTi ILC3s is able to trigger the formation of ectopic lymphoid aggregates in inflamed tissue sites and thereby influence the quality of the mucosal immune response (224). Besides their impact on the induction of ectopic lymphoid aggregates, ILC3s might further contribute to the recruitment of ILCs to local sites of inflammation via the release of GM-CSF. A study conducted by Pearson et al. (227) identified circulating and colon-infiltrating ILC3s as a relevant source of GM-CSF in humans and described a significant upregulation of GM-CSF^+^ ILC3s in the blood of IBD patients. Based on observations in murine colitis, the inflammation-triggered exit of ILCs from colonic cryptopatches into the adjacent tissue is GM-CSF-dependent and can thus be promoted by activated ILC3s (227). However, this functional link between ILC3-derived GM-CSF and innate immune cell mobilization from ectopic lymphoid aggregates still needs to be confirmed for the human system.

Taken together, more intense research is necessary to validate our current understanding of the systemic and local mobility of human ILCs, as it is still mainly based on phenotypical observations and *in vitro* findings. Most likely, the availability of humanized mouse models will substantially support us in achieving new insights into the chemotactic stimuli attracting blood ILCs under various *in vivo* pathophysiological conditions. Since our current knowledge of chemotactic ILC attraction has been mainly restricted to ILC2s, upcoming analyses should also include research into the migratory capacity of ILC1s and ILC3s.

## Clinical Implications

Even though ILC activity is controlled by a tight regulatory network within the human body, dysbalanced ILC frequencies and activity have been observed in the context of numerous diseases characterized by chronic inflammation, fibrosis, or malignant transformation of mucosal tissues (15, 60, 146, 228). Due to their remarkably fast and potent capacity to react to stress signals with the release of immune coordinating effector cytokines, ILCs might represent important target structures for innovative biomarker and treatment strategies. Although our knowledge of ILCs has grown exponentially in the last decade, no ILC-specific application has yet entered the clinics. However, the therapeutic efficacy of several T cell-targeting standard therapies might actually derive from their combined suppressive effects on T cells and ILCs. For instance, glucocorticoid therapy was able to normalize enhanced blood ILC2 frequencies in asthmatic patients (229). Since ILC2s have been suggested to be the main producers of the pro-inflammatory cytokines IL-5, IL-9, and IL-13 in asthmatic patients (229), their contribution to pathologies must not be underestimated. Similarly, systemic glucocorticoid treatment reduced nasal ILC2 proportions in patients with eosinophilic nasal polyps (230). In accordance with these *in vivo* observations, *in vitro* studies confirmed a direct inhibitory effect of the glucocorticoids dexamethasone and budesonide on the cytokine production of activated human blood ILC2s (83, 229, 231), which were proven to express the glucocorticoid receptor (229). Interestingly, this dexamethasone responsiveness turned out to be dependent on the stimuli activating ILC2s. While IL-25- and IL-33-driven ILC2 activities could be successfully suppressed by dexamethasone, this was not the case for IL-7- and TSLP-stimulated human blood ILC2s (231). In line with this, BAL ILC2s derived from asthmatic patients that had been exposed to elevated TSLP levels *in vivo* also displayed dexamethasone resistance (231). Given the elevated levels of both IL-33 and TSLP in the BAL of asthmatic patients (232), the therapeutic efficacy of glucocorticoids might largely depend on the inflammatory microenvironment.

Another commonly used drug in the therapy of asthma, the leukotriene receptor 1 antagonist montelukast (233), is known to relevantly impact the fate of ILC2s. Based on its inhibitory effect on the cytokine production of human skin and blood ILC2s *in vitro* (87, 89), it is reasonable to assume that the *in vivo* efficacy of montelukast is also supported by its ILC2-dampening capacity. In cultured ILC2s, montelukast could further be proven to abrogate the chemotactic and anti-apoptotic potential of cysteinyl leukotrienes (89).

More recently, anti-cytokine therapies have been successfully introduced in the treatment of various inflammatory diseases and partly also target important ILC effector cytokines. For instance, patients with severe nasal polyps showed significantly decreased disease severity upon treatment with the anti-IL-5 antibody mepolizumab (234). Moreover, beneficial effects of anti-IL-4 and anti-IL-13 antibodies have been suggested for a subgroup of asthmatic patients (235, 236). These data strongly imply that treatments originally designed to target T cells and their effector cytokines might additionally function by modifying ILCs. Whether ILCs can also be targeted specifically is unclear to date and requires further research. Based on our current knowledge, however, the partial functional redundancy between ILCs and Th cells under physiological conditions (26) and the crucial impact of mucosal ILCs on multiple inflammatory disorders (6, 75) qualifies this innate cell type as an excellent therapeutic target with minimal adverse events (5, 237).

## Conclusion

While the explicit benefit of ILCs for healthy individuals has been questioned under the very high hygiene standards in industrialized countries (26), ILCs have been impressively proven to play essential roles in multiple pathologies. In particular, their prime function as guardians and first line of defense at mucosal barrier surfaces makes them a key factor deciding between the induction of controlled and protective or overwhelming and detrimental immune responses upon pathogen entry. Thus, a tight regulation of ILC numbers and their activity is highly important. Indeed, a dense network has been identified that regulates human ILCs, consisting of soluble factors as well as cell contact-dependent processes. These mediators can directly regulate the activity of local ILCs but can also adapt tissue-resident ILC numbers by modulating the viability and proliferative capacity of local ILCs and their potential for transdifferentiation. Moreover, ILCs can be redistributed within an organ or recruited from distal sites to adjust the ILC pool within inflammatory tissue sites according to local requirements. Albeit controversial, homing of human blood ILCs to the site of action represents an interesting, yet underrated phenomenon that requires further analysis (Figure 1). Even though enormous progress has been made regarding our knowledge of human ILC regulation, until now, this is largely based on *in vitro* experiments. Human *in vivo* data are, however, mainly restricted to association studies. These have successfully identified great correlations of ILC frequencies with chronic lung and gut inflammation but lack functional evidence. Meanwhile, *in vivo* studies have been primarily conducted on murine ILCs, and translation of functional results to the human system often remains unsatisfying. Therefore, future studies might reinforce the use of humanized mouse models in ILC research. This might allow the central question of whether altered ILC frequencies in disease are cause or consequence to be tackled, which is particularly important with regard to the potential development of ILC-targeting therapeutic strategies. Until ILCs can be used therapeutically, however, many gaps have to be filled, and our understanding of human ILCs has to be expanded significantly. Therefore, larger patient cohorts should be examined in combination with sophisticated *in vitro* and *in vivo* analyses. Overall, a crucial role of ILCs in mucosal immunity has been impressively determined in the last decade, making the analysis of the functional contribution of human ILCs to fibro-inflammatory diseases and their potential therapeutic modulation a central target for the next 10 years.

## Author Contributions

AS-K, SW, MN, and IA drafted and wrote the manuscript. All authors contributed to the article and approved the submitted version.

## Conflict of Interest

The authors declare that the research was conducted in the absence of any commercial or financial relationships that could be construed as a potential conflict of interest.
